# The Risk Model of Traffic Engineering Investment and Financing by Artificial Intelligence

**DOI:** 10.1155/2022/9402472

**Published:** 2022-08-03

**Authors:** Shangen Wang, Wei Zhang

**Affiliations:** ^1^School of Management Engineering, Zhengzhou University, Zhengzhou, Henan 450001, China; ^2^School of Management, Shanghai University, Shanghai 200444, China

## Abstract

This study aims to analyze the influencing factors and mechanisms of investment and financing risks in transportation projects so that regions do not restrict the transportation investment and financing risk models in all areas to achieve intelligent transportation financial risk assessment. Firstly, the investment and financing modes are studied and analyzed. According to the analysis of intellectual investment and the financing report of traffic engineering infrastructure, a traffic engineering investment and a financing model based on intelligent computing is established, which is based on artificial intelligence (AI) big data analysis technology. Secondly, the investment and the financing risk model of traffic engineering is established based on multimodal learning. Finally, the urban traffic engineering of Xi'an is taken as the research object. Based on its investment and financing data in the construction of urban roads, the risk assessment is carried out. Combined with risk influencing factors, the accuracy of the intelligent calculation in the risk assessment model is calculated. Different grades of urban transportation projects have different risks in the investment and financing of transportation projects. The results show that different levels of urban transport projects have different risks in the investment and financing (IAF) performance of transport projects. Among them, the risk index of the first-class project is the highest, reaching 0.55. The risk index of the second-class project is 0.49. The results before and after using the flow engineering IAF risk model are compared. In the test results of traffic engineering risk, all target risks did not increase after the AI-based traffic engineering IAF is tested. The model test results for credit risk and financial risk are the highest at 70 and 60, respectively. Combined with the actual urban development situation, this study can provide investment and financing risk models for urban transportation projects in different regions and provide a reference for the resource control of transportation projects. This study uses AI to learn and analyze traffic engineering investment and financing data and more accurately provide data references for traffic engineering investment and financing risk models.

## 1. Introduction

In recent years, discipline inspection and supervision organs of Shaanxi province have thoroughly implemented the decision and deployment of the 19th CPC National Congress on strengthening anti-corruption efforts in the financial field, preventing and resolving major financial risks, and closely focused on government investment and financing (IAF) platforms, and seriously investigated and punished some serious violations of discipline and law by the principals. Additionally, the procuratorial organs maintain a high-pressure attitude of punishing bribery and seriously investigate and punish bribery, forming a strong deterrent [1, 2]. As the economic entity that mainly undertakes the financing function of government-invested projects, IAF platform companies are the “rich area” where public resources such as capital, land, and equity are relatively concentrated, and the “high incidence area” of illegal financing guarantee, illegal borrowing, and illegal borrowing investment. Corruption in the field of IAF will not only cause huge losses of state-owned assets and increase the risk of government IAF but also lead to serious consequences, such as hidden dangers in the quality of public construction projects, deterioration of the business environment, and damage to the political ecology [3, 4]. The *Outline for Building a Strong Transportation Country* proposes to “strengthen financial security, deepen the reform of transportation IAF, enhance sustainable development capabilities, and improve a government-led hierarchically responsible for diversified financing, risk-controllable capital security, and operation management system.” The document proposes to “establish and improve the financial investment guarantee system at all levels at the central and local levels, encourage the use of diversified market financing methods to expand financing channels, actively guide social capital to participate in the construction of a strong transportation country, and strengthen the construction of risk prevention and control mechanisms” [5]. The IAF business of transportation planning is closely related to the city scale, layout form, road network structure, and economic level. The urban transportation planning and design unit where the project is located has relatively rich experience and performance in territorial projects. Additionally, a database related to territorial traffic and urban construction can be established. The database has a strong advantage in the process of business competition [6–8].

Li and Love studied the economic risks of the public-private partnership (PPP) model of urban transit rail engineering projects. The traffic of Beijing metro line 4 is used as the research object. In transportation projects, the relevant analysis of economic risks such as subway fares, people flow, subway operating costs, and relevant government subsidies are analyzed. According to different economic risks, corresponding opinions are put forward [9]. Wang et al. analyzed the application of the PPP model in Sichuan. They mainly studied the application of this model in public services in Sichuan. In these public service applications, the government has a dominant position in the achievement of the PPP model [10]. However, because the PPP mode templates are different, the operating mechanisms in different regions are also different. Chang and Su took the Australian PPP project as the object and analyzed the implementation process and the preassessment system of the project. Based on the situation of China's preassessment of PPP projects, they summarized a new path for the development of PPP projects [11]. Owusu-Manu et al. studied the asset securitization financing model for transportation and rail projects. Guangzhou Nansha transportation rail was taken as the research object. They analyzed the feasibility of the asset securitization financing model and designed a financing plan. Scholars put forward the corresponding measures to deal with the asset securitization risk in the financing process [12]. Liu et al. used quantitative research to promote the implementation of asset securitization based on the existing problems of asset securitization in PPP projects [13]. Bai and Zhang optimized the transaction structure of asset-backed PPP projects. The optimization results can not only enhance the liquidity of the assets of the trading standard through the expansion of the trading platform but also attract investors to participate in asset securitization and promote the application of asset securitization [14]. The extensive application of artificial intelligence (AI) technology in the field of transportation engineering under asset support has a practical application value for the development of real assets.

In order to analyze the influencing factors and mechanism of IAF risk of transportation projects, the transportation IAF risk model of each region is not limited by the region. The assessment of transportation financial risks is intelligent [15, 16]. Firstly, the IAF patterns of traffic engineering are analyzed. The innovation lies in intelligent IAF report analysis based on traffic engineering infrastructure and based on AI big data analysis technology. A traffic engineering IAF model based on intelligent computing is established. The expected result is to use multimodal learning to build a transport project IAF risk model. Finally, the urban traffic engineering of Xi'an is taken as the object. According to IAF, data on urban road construction are subjected to risk assessment. Combined with risk influencing factors, the accuracy of the intelligent calculation in the risk assessment model is analyzed. The disadvantage is that the accuracy of the algorithm's intelligent calculation needs to be further improved. This study has practical application value for investment and financing financial risk estimation in transportation engineering.

## 2. Establishment of Different Risk Models for Traffic Engineering

### 2.1. IAF Mode of Transportation Engineering

There are various types of rail transportation, such as subway, light rail, suburban railway, ghost tram, and maglev train. In September 2019, the *Outline for Building a Strong Transportation Country* issued by the Central Committee of the Communist Party of China and the State Council proposed to reform the current investment and the financing system for transportation projects. The document mentions that it is necessary to strengthen capital guarantee, deepen the reform of transportation financing, enhance the ability of sustainable development, and improve the capital guarantee and operation management system led by the government, responsible for different levels, diversified financing, and controllable risks. Financial input guarantee systems at the central and local levels should be established and improved. The government encourages the use of diversified market financing methods to expand financing channels, actively guides social capital to construct a strong transportation country, and strengthens the construction of risk prevention and control mechanisms. The promulgation of this document puts forward new requirements for the IAF mode of traffic engineering. The IAF methods of transportation projects are shown in Figure 1.

In Figure 1, government-issued bonds include the bonds issued by the central government and general securities and special bonds issued by local governments. Public-private partnership (PPP) is a competitive way for governments to select private partners with investment, operation, and management capabilities. The two parties sign a contract after equal negotiation, clarifying the relationship between responsibilities and rights. Social capital provides public services, and the government considers social capital based on the results of public interest evaluation to ensure that social capital obtains a reasonable return [17]. Figure 1 shows the IAF transport engineering model of transport. The IAF system of transportation engineering is shown in Table 1.

The government dominates the traditional IAF model. In addition to the government's direct investment in construction, it also includes government debt and government-guaranteed financing. Project construction is carried out by issuing government bonds or borrowing directly from banks by the government. Under the market-oriented IAF model, enterprises aim to obtain profits. Corporate credit or project proceeds are used to raise funds for project construction using commercial financings such as commercial loans and the issuance of bonds and stocks. In terms of financing entities, its IAF models mainly include build-transfer (BT), PPP, and build-operate-transfer (BOT). PPP is a project operation model in public infrastructure. This model encourages private enterprises, private capital, and the government to cooperate and participate in the construction of public infrastructure. PPP refers to that in the public service. The government selects social capital with investment and operation management capabilities competitively. The two parties conclude contracts under the principle of equal consultation. The social capital provides public services, and the government considers the social capital based on the performance evaluation results of the public service. PPP provides services in market competition, mainly in the pure and quasi-public domains. PPP is not only a financing method but also a system and mechanism reform involving administrative, financial, and IAF system reform [18]. The PPP model is shown in Figure 2.

In Figure 2, the PPP model is an optimized project financing and implementation model. The “win-win” or “multi-win” of each participant is the basic concept of cooperation. The essence of this form of financing is that the government accelerates infrastructure construction and efficient operations by granting long-term franchise and revenue rights to private companies. As a new project financing model, PPP ensures the “profitability” of private capital to a certain extent. This model can attract private investment to the maximum extent, allow more private capital to participate in the project, and reduce the pressure on government investment capital. PPP reduces government debt, transforms government departments from infrastructure public service providers to regulators, supervises and manages the construction and operation of public products, supervises the quality of transportation products, makes them safer, and promotes the transformation of government functions. Project sponsors select suitable private partners in a fair, open, and competitive manner. They can improve the construction and operation efficiency of rail transit, reduce project costs, and reduce overall government costs and subsidies. Project investors can also achieve profit returns in vehicles, mechanical and electrical equipment, rail engineering construction, etc., and strictly control costs by strengthening management.

The BOT model means that the government department signs a concession agreement with a private enterprise (project company) on an infrastructure project and grants the contracted private enterprise (including foreign enterprises) to undertake the investment, financing, construction, and maintenance. During the concession period specified in the agreement, the model allows it to finance the construction and operation of specific public infrastructure and repay the loan by charging users fees or selling products, recovering investment, and earning profits. The government has the power to monitor and manage this infrastructure. At the expiry of the concession period, the private sector of the contracting party will hand over the infrastructure to the government for free or for a fee. Under the BOT model, investors usually ask the government to guarantee their minimum rate of return. If the standard cannot be met within the concession period, the government shall pay special compensation. BOT has the characteristics of a mixed economy combining market mechanisms and government intervention. According to the way of investment and financing of transportation projects, it is necessary to realize the ideal combination in its source (bond or loan, etc.), interest rate (fixed or floating), financing preparation time, repayment period, currency, etc., so as to determine the allowable investment and financing risk index. The Hong Kong MTR Corporation has formulated an “ideal financing model.” The model summarizes important financing and risk management strategies and identifies corresponding metrics. The IAF structure is optimized from the four dimensions of capital source, interest rate type, loan term, and financing currency. The financing cost and financing risk are effectively controlled [19].

In summary, several traffic engineering models have in common that they can provide strategies for financial risk estimation. The advantage of the IAF model lies in government leadership and financing. The advantage of the PPP model is that the government is a new financing model by granting long-term franchise and income rights to private companies. The BOT model allows it to finance the construction and operation of specific public infrastructure. The government has the power to monitor and manage these infrastructures. The ideal IAF model is shown in Table 2.

### 2.2. AI and Back Propagation Neural Network

Today, AI technology has penetrated all walks of life, not only creating new industries and new formats but also bringing vitality to traditional industries. In the past, the concept of AI was more combined with applications, such as face recognition and machine recognition. Today, AI will help the economic field of transportation engineering from three aspects: prediction, monitoring, and optimization. This is due to the advantages of AI technology in computing power. These advantages are due to the digital needs of all walks of life. By providing lower-cost and more efficient innovative solutions in the digital industry, serving enterprises will become a long-term gold nugget field. The operation mechanism of AI is shown in Figure 3.

In Figure 3, AI is divided into strong and weak. Strong AI uses computers to construct complex machines with the same essential characteristics as human intelligence. This study uses the back propagation neural network (BPNN) algorithm to learn the IAF risk model of traffic engineering, reduce the prediction risk error, and improve the prediction accuracy of IAF risk. The network structure of the BPNN algorithm is shown in Figure 4.

In Figure 4, the BPNN algorithm is a multilayer feedforward neural network trained according to the error back-propagation algorithm and given an input vector. The output is obtained in a single forward pass [20, 21]. The BPNN algorithm is employed for 1000 model iterations, consisting of inputs, weights, and outputs. The algorithm training data set adopts the MNIST handwriting data set. Different grid parameters are used to train and study the model. The input to net_*j*_ is *X*. The weight *V* is utilized to obtain the output *O*=(*o*_1_, *o*_2_,…, *o*_*i*_,…, *o*_*n*_). The weight parameters from the input layer to the hidden layer are *V* and *W*. The input calculation expression of the *h*th hidden layer neuron is shown in equations (1) and (2):

(1) $$\begin{array}{c} {\text{net}}_{j}=\sum_{i=1}^{n}v_{ih}x_{i}, \end{array}$$

(2) $$\begin{array}{c} y_{j}=f\left({\text{net}}_{j}-\theta_{j}\right), \end{array}$$

where *x*_*i*_ represents the input to the *i*th neuron. *n* is the number of neurons and the net input net_*j*_ of the neuron is obtained by linear weighted summation. *v*_*ih*_ is the weight from the input layer to the hidden layer. *θ*_*j*_ is the threshold of this neuron. *f* is the selected activation function. Similarly, the net input and actual output of the neurons in the output layer can be derived. A gradient descent strategy is adopted. The target negative gradient direction is used to update the parameters. The learning rate *ηϵ*(0,1) is given. The sigmoid activation function is chosen to transform each net_*j*_ regression value. Its derivative properties are shown in equation (3):

(3) $$\begin{array}{c} f^{\prime }\left(x\right)=f\left(x\right)\left(1-f\left(x\right)\right). \end{array}$$

The output value of each node is based on the output values of all nodes in the upper layer. The weights of the current node and all nodes in the previous layer and the threshold and activation function are implemented. In Figure 5, the calculation expression of the output value of node *k* is shown in equations (4) and (5):

(4) $$\begin{array}{c} {\text{net}}_{k}=\sum_{i=0}^{I}W_{ik}*X_{i}, \end{array}$$

(5) $$\begin{array}{c} O_{k}=f\left({\text{net}}_{k}-B_{k}\right), \end{array}$$

where *B*_*k*_ is the threshold of the *k*th neuron in the hidden layer; *W*_*ik*_ is the weight from the hidden layer to the output layer; *f* is the activation function, according to equations (4) and (5), the forward propagation ends from the input layer to the hidden layer to the output layer. In the output layer of BPNN, the error calculation expression between the output result of the input data processed by the network and the standard result is shown in equations (6) and (7):

(6) $$\begin{array}{c} E=\sum_{k=1}^{m}E_{k}, \end{array}$$

(7) $$\begin{array}{c} E_{k}=\frac{1}{2}\sum_{i=1}^{n}\left(y_{ik}-{\hat{y}}_{ik}\right)=\frac{1}{2}\sum_{i=1}^{n}\delta_{o}^{2}. \end{array}$$

Equation (5) is a sum-of-squares performance index function based on the gradient method to minimize the sum-of-squares performance index function. *m* is the number of samples; *E*_*k*_ is the local error function. *y*_*ik*_, ${\hat{y}}_{ik}$ are the expected output and the actual output of the *k*th learning mode, respectively; *δ*_*o*_ is the deviation between the expected output and the actual output. In the same way, *δ*_*y*_ and *δ*_*y*_ are calculated as the deviation between the expected input and the actual input. The calculation of weight adjustment is shown in equations (8) and (9):

(8) $$\begin{array}{c} \Delta V_{ij}=-\eta \frac{\partial E}{\partial V_{ij}}, \end{array}$$

(9) $$\begin{array}{c} \Delta W_{ij}=-\eta \frac{\partial E}{\partial W_{ij}}. \end{array}$$

The delta learning rule is used to change the connection weights between neurons to reduce the error between the actual output and the expected output of the system. The number of nodes in the input and output layer is determined. The number of nodes in the hidden layer impacts the training performance of the BP algorithm. Equation (10) is used to determine the number of hidden layer nodes:

(10) $$\begin{array}{c} h=\sqrt{n+m}+\alpha . \end{array}$$

In equation (10), *h* is the number of hidden layer nodes; *n* is the number of input layer nodes; *m* is the number of output layer nodes; *α* is an adjustment constant between 1 and 10. During the training process, the BP algorithm can easily form a local minimum and cannot obtain an optimal global value. The increase in training times leads to low learning efficiency and slow convergence speed. The algorithm is improved to avoid these problems. The momentum term to accelerate algorithm convergence is introduced, as shown in the following equation:

(11) $$\begin{array}{c} \Delta w_{ij}\left(t+1\right)=\eta \delta_{y}x_{i}+\gamma \Delta w_{ij}\left(t\right). \end{array}$$

In equation (11), Δ*w*_*ij*_(*t*+1) represents the variable that connects the weights of input nodes *x*_*i*_ and *x*_*j*_ at time *t*+1. *η* is the learning rate; *γ* is the momentum factor *γ*∈[0.1, 0.8]; *δ*_*y*_ is the error of the input node *x*_*i*_. Adaptive adjustment of the learning rate or the steepness factor is introduced for algorithm improvement.

### 2.3. Establishment of the Traffic Engineering IAF Risk Model

Based on the existing traffic engineering, IAF operating mechanism, and multimodal learning, a model of traffic engineering IAF risk is established. Multimodal learning can establish the risk model of traffic engineering IAF. The machine learns the information of each modal and realizes the exchange and conversion of information [22]. When the BPNN algorithm is used for intelligent calculation of the training process, an attention mechanism is introduced, and an attention alignment model is established. The alignment model consists of two layers of neurons to form a neural network, and the output representation is shown in the following equation:

(12) $$\begin{array}{c} e_{ij}=a\left(s_{i-1},h_{j}\right)=v_{a}^{T}\text{tanh}\left(W_{a}s_{l-1}+U_{a}h_{j}\right). \end{array}$$

In equation (12), *W*_*a*_, *U*_*a*_ and *v*_*a*_ are the weight matrix; *T* is the length of the input traffic engineering IAF information; *h*_*j*_ is the hidden variable at time *j*; *s*_*i*−1_ is the implicit variable of output investment and financing data in the BP network for the decoder; *e*_*ij*_ is the energy value of the correlation between the data output of each IAF data and the predicted IAF risk. The IAF risk model of traffic engineering is shown in Figure 5.

## 3. Results Analysis

### 3.1. Risk Analysis of IAF of Urban Traffic Engineering at Different Levels

The urban traffic engineering of the Xi'an city is taken as the object. IAF data in the construction of urban roads are subject to risk assessment. According to the *Interim Provisions on Urban Planning Quota Indicators*, urban traffic engineering in Xi'an is divided into four grades. The first-level projects are generally connected to important economic, political, and cultural centers and traffic projects at some interchanges; the second-level projects are trunk roads connecting political and economic centers or suburban traffic projects with heavy traffic; tertiary projects are feeder traffic projects connecting cities at or above the county level; grade IV projects refer to feeder traffic projects connecting counties, towns, and townships. The IAF risk analysis of different levels of urban transportation projects is shown in Figure 6.

In Figure 6, different levels of urban transport projects have different risks in the IAF performance of transport projects. The risk index of the first-level project is the highest, which is 0.55. The risk index of the second-level project is 0.49. The risk index of the third-level and fourth-level projects is 0.34 and 0.21, respectively. The higher the level of flow engineering, the higher the financing risk. The rating is closely related to the economic environment, government support, land use, and other influencing factors of the actual traffic IAF. The actual risk index is not much different from the prediction, indicating that the flow engineering IAF risk results simulated by the established model are consistent with the actual value, and the model fits well.

### 3.2. Analysis of Test Results of the Traffic Engineering IAF Risk Model

According to the influencing factors of IAF risks of transportation projects, the target risks are divided into seven kinds of tests to analyze the accuracy of the intelligent calculation in the risk assessment model, namely social, policy, credit, credit, construction, operational, and financial risks. The test of the risk model of traffic engineering IAF is shown in Figure 7.

In Figure 7, the results before and after using the traffic engineering IAF risk model are compared. From the test results of traffic engineering risks, after the IAF test of traffic engineering based on AI is adopted, all target risks have not increased. Policy and social risk do not change significantly before and after the model is used. Predictions of credit, construction, operations, and financial risks have significantly weakened. This conclusion shows that the designed model has a little effect on predicting irresistible IAF risks. The designed model can reduce IAF risks.

To sum up, the IAF risk model of traffic engineering AI is established. Xi'an urban traffic engineering is taken as the research object. According to the risk assessment of its IAF data in urban road construction, the higher the level of the transportation project, the higher the IAF risk it undertakes. All target risks are not increased after the AI-based IAF is tested. Policy and social risks do not change significantly before and after model use. In addition, the results of this study are compared with other studies. Luo et al. [23] researched SME investment and financing under the public-private partnership model. By comparing with pure private borrowing, they found that silver-tax interaction can make investment cheaper and more attractive, alleviating the problem of underinvestment in volatile markets. Sarkar and Zhang [24] researched corporate investment and financing decisions. The results showed that leverage has a positive effect on overall investment. The difference between leveraged and unleveraged firms is an increasing learning rate function. The optimal leverage ratio (without borrowing constraints) is an increasing learning rate function. Koohkan et al. [25] studied the influencing factors of corporate investment and financing decisions. The results showed that investors' psychological accounting has a significant adverse effect on financial leverage and cash dividends and has a direct impact on debt ratio, debt maturity, and long-term debt-equity ratio as indicators of corporate financing policy. In addition, investor psychology can adversely affect changes in tangible fixed assets, which are corporate indicators. Therefore, the proposed IAF can achieve higher risk assessment accuracy at a lower risk.

## 4. Conclusion

This study aims to ensure that the transportation project of IAF marketization and sustainability, accurate positioning support the national major strategic implementation of major transportation projects, to increase the intensity of support further, improve service levels, strengthen risk control, distinguish between different regions, different types of financing. The research can provide strong financial support for the construction of a powerful transportation country. It provides a risk reference for the sustainable development of the transportation engineering economy. The model established by the research is not limited by the regional scope and can provide the IAF risk model for urban transportation projects in different regions and provide a reference for the resource control of transportation projects. This study uses AI to learn and analyze traffic engineering IAF data and more accurately provide data references for traffic engineering IAF risk models. However, the established traffic engineering IAF risk model involves too many influencing factors. Therefore, the model still has some shortcomings. The main disadvantage is that many people participate in the system according to the IAF risk of traffic engineering projects. While pursuing the maximization of traffic engineering benefits, they also need to avoid losses caused by risks. Based on the game theory, this study designs a risk-sharing scheme for IAF risks of transportation projects to reduce financing risks.

## Figures and Tables

**Figure 1:** The way of IAF of traffic engineering.

**Figure 2:** PPP mode.

**Figure 3:** The working mechanism of AI.

**Figure 4:** Network structure of the BPNN algorithm.

**Figure 5:** Risk model for IAF of transportation engineering.

**Figure 6:** Risk analysis of IAF of urban traffic engineering at different levels.

**Figure 7:** Analysis of the test results of the IAF risk model of traffic engineering.

**Table 1:** The system of IAF for transportation projects.

Financing system	Financing subject	Financing model
Government financing model	An economic entity with legal personality and authorized by the government to engage in financing activities	Operation and management of government administrative agencies, operation, and management of corporatized entities
Commercial financing model	Taking enterprises as the main body of investment in projects	Corporate credit financing and project financing
Blend mode	Government-invested, nonproprietary sole proprietorship company	For example, the PPP mode

**Table 2:** Ideal IAF model.

Project	Ideal financing model	Actual debt structure
Capital market tools	50%∼80%	79%
Medium-term loan	20%∼50%	16%
Export credit	0∼10%	1%
Short-term loans and bank overdrafts	0∼15%	4%
Fixed-rate	40%∼60%	61%
Floating rate	40%∼60%	39%
Financing preparation period	6 to 15 months	12 months
Repayment period within two years	10%∼40%	15%
Repayment period 2∼5 years	20%∼50%	48%
Repayment period after 5 years	30%∼60%	37%
Hong Kong dollar	70%∼100%	99.8%
Dollar	0∼30%	0.2%

Data source: Hong Kong MTR Corporation.

## Data Availability

The dataset used in this paper is available from the corresponding author upon request.
